This article has been retracted.

# Characteristics of Aerobics and Nutrition Strategy Based on Depth Image Human Body Recognition

**DOI:** 10.1155/2022/8021536

**Published:** 2022-02-08

**Authors:** Liangliang Cheng, Dongfang Nie

**Affiliations:** Department of Sports, Chongqing University of Science and Technology, Chongqing 401331, China

## Abstract

Bodybuilding operation is a favorite sports item, which is beneficial to enhance physical fitness, improve coordination and flexibility of movement, and enhance cardiopulmonary function. Standard aerobics movements and nutrition matching strategies can more effectively enhance the exercise effect. In this paper, the characteristics of aerobics, sports, and nutrition strategies are researched through the human body recognition technology of the depth image; the subjects were divided into four groups by statistical method and control variable experiment method. They were the control group, the experimental group for aerobics training, the experimental group for improving the nutritional balance under diet, and the experimental group for aerobics training. After two and a half months of experimental training and observation, the students in the four groups were tested for physical fitness and physical function; analyze the obtained experimental test data using the human body recognition technology of depth image, then obtain the experimental test data, and then use the data fusion method to combine the data and information for more accurate evaluation. The results showed that after 10 weeks of aerobics learning and nutrition, the average height of students increased by 1.19 cm, the average weight decreased by 1.17 kg, the number of sit-ups increased from 23.9 before the experiment to 31.2, and the results of 50-meter race and 800-meter run were 0.2 seconds and 2.9 seconds, respectively. It can be concluded that aerobics and nutrition can speed up metabolism, promote the growth and development of bones, and supplement the nutrition needed by the human body, to improve students' physical quality. This study contributes to the research of sports and nutrition matching in improving physical conditions.

## 1. Introduction

In recent years, a variety of media often appear to worry about the physical strength of young people. Among them, obesity and malnutrition are the most significant factors threatening the health of young people. If the physical health problems of teenagers are not effectively improved, it will threaten their future health and greatly reduce their quality of life. From a social point of view, this will also greatly increase the future of national health care. For health insurance and pension fund expenditure and national construction, this is also an obstacle to talent training strategy. Human action and behavior recognition has always been a hot research topic in multiple crosscutting fields such as computer vision and pattern recognition. It has broad application prospects such as human-computer interaction, smart home, and smart monitoring.

As a hope for the future development of society, young students should not only pay attention to the effectiveness of students' learning but also pay attention to the growth state and shape of their bodies. Therefore, the use of effective sports and nutrition to improve students' physical strength is the key to the healthy growth of students. Regular and planned exercise can improve students' cardiopulmonary function, strengthen their muscles and bones, and maintain smooth blood circulation, to realize the effective development of body metabolic function. Moreover, through the use of appropriate nutrition, maintain daily intake of vitamins, protein, and sugar; make an excellent diet to improve body immune structure; strengthen disease prevention ability; improve students' immunity; and achieve the goal of maintaining health. Aerobics exercises are very helpful for improving physical fitness and shaping the body. It can thicken muscle fibers with various intensities of muscle activity, thereby achieving the purpose of shaping the body. At the same time, exercise load stimulates internal organs, promotes breathing, accelerates blood circulation, improves nervous system function, strengthens the body's immunity, and ensures youth's health. As for physical health and quality of life, the most important thing is that there have been earlier studies on the physical health of young people abroad, but domestic research has not been particularly in-depth, so it is essential to carry out research on it now.

In the study of aerobics training and nutrition balance, Hoelscher et al.'s research is aimed at showing the preliminary results of the implementation of futp60 in 72 schools of grades 6-9. His study used noncontrolled pretest/posttest and continuous cross-sectional data. School health practices were documented during the baseline needs assessment survey [1]. Basso-Vanelli et al.'s study was performed to compare the effects of inhalation muscle training, aerobics, and physical exercise-related breathing exercises on COPD subjects as additional benefits of inspiratory muscle strength and endurance, chest and abdominal exercise ability, physical exercise ability, and reduction of exertional dyspnea. Their study also compared these gain weaknesses in subjects with and without respiratory muscles. Their method has a certain effect, but the stability is poor [2].

In this study, the control variable method was used to divide the subjects into four groups. After that, the students were tested, including standing, long jump, 50 m, 800 m, height, weight, sebum thickness, vital capacity, and step test. Deep image human body recognition technology was used to recognize and analyze the movements of aerobics, improve people's aerobics movements, and make them more standard. Through data fusion, data and information are combined for more accurate evaluation. Analysis of the effects of aerobics training and nutritional collocation on the results of the experiment on the physical indicators of students, on students' physical quality index, on students' daily diet and nutritional status, and on students' comprehensive physical quality was performed. The main innovation is to use deep image human body recognition technology to recognize and analyze aerobics movements, improve people's aerobics movements, and make them more standardized [3, 4].

## 2. Human Body Recognition Technology of the Depth Image Matches the Characteristics of Aerobics with the Physical Nutrition of the Students

### 2.1. Human Body Recognition Technology Based on Depth Images

Visual analysis of human motion has been a hot topic in recent years and has attracted much attention in the field of machine vision. It has broad application prospects and potential economic value in the fields of human-computer interaction, video conferencing, medical diagnosis, game animation, virtual reality, and security monitoring of communities, supermarkets, banks, and image storage, which has attracted researchers and related companies of great interest. Human contour recognition is an important part of human motion visual analysis [5]. The accuracy of recognition will directly affect the success of human motion visual analysis, so it has important theoretical value and a wide range of applications. Traditional human contour recognition technology is mainly based on RGB color images taken by visible light cameras, which is not robust. The main reason is that it is easily affected by factors such as light changes, complex environments, and object occlusion. The goal of human motion recognition is to automatically detect and analyze human behavior from video data. The data source can be an image sequence obtained from an RGB camera, a distance sensor, or other mode sensors. In sports competition, we can get the standard action template of the project through video analysis of a large number of sports competitions. In the daily exercise of aerobics, the executive action is compared with the template to determine the shortcomings of oneself or correct the mistakes of the action. Visual information is embodied in the fields of computer vision and pattern recognition as the processing, analysis, learning, and understanding of the content of images or videos. Among them, the detection and tracking of moving targets in video, especially the detection of human bodies and the analysis and recognition of individual actions, have important academic value. This helps us to deeply understand the human body's movements, to carry out higher-level behavior analysis and recognition.

### 2.2. Data Fusion

Data fusion refers to the process of using computer technology to process information under specific standards. The process can automatically analyze, optimize, and integrate sensor observations that require sufficient time to complete the required decision-making and evaluation tasks. Data fusion is also called information fusion or multisensor fusion, the process of using computer technology to process information under certain conditions. This process can automatically analyze, optimize, and synthesize time series multisensor observations to complete the required set of decision-making and evaluation tasks. With the continuous development of science and technology, the data environment in future life will become more complex, and the amount of data will increase exponentially. At the same time, there is still a lot of uncertain and false information. In this case, the continuous development of data fusion technology will significantly improve the efficiency of information processing and provide accurate, timely, and effective information support for data decision-making.

The Kalman filter (KF) algorithm is actually an application of the “estimation” idea. “Estimation,” in short, is to extract effective information from observations that contain errors. The algorithm flow is shown in Figure 1.

Ignoring the control effect of the system, the equation of the stochastic linear discrete system can be expressed as

(1) $$\begin{array}{c} \left\{\begin{array}{c} Xk=\phi_{k,k-1}X_{k-1}+\tau_{k,k-1}W_{k-1},\\ Z_{k}=H_{k}X_{k}+V_{k}. \end{array}\right. \end{array}$$

It is assumed that the process and observation noise of the system have the following characteristics:

(2) $$\begin{array}{c} \left\{\begin{array}{c} E\left[W_{k}\right]=0,E\left[W_{k}{W_{j}}^{T}\right]=Q_{k}\delta_{kj},\\ E\left[V_{k}\right]=0,E\left[V_{k}{W_{j}}^{T}\right]=R_{k}\delta_{kj},\\ E\left[W_{k}{W_{j}}^{T}\right]=0. \end{array}\right. \end{array}$$

One-step state prediction equation

(3) $$\begin{array}{c} {\hat{X}}_{k,k-1}=\phi_{k,k-1}{\hat{X}}_{k-1}. \end{array}$$

State estimation equation

(4) $$\begin{array}{c} {\hat{X}}_{k}={\hat{X}}_{k,k-1}+K_{k}\left[Z_{k}-Z_{k,k-1}\right],\\ {\hat{Z}}_{k,k-1}=H_{k}X_{k,k-1}. \end{array}$$

Filter gain matrix

(5) $$\begin{array}{c} K_{k}=P_{k,k-1}{H_{k}}^{T}{\left[H_{k}P_{k,k-1}{H_{k}}^{T}+R_{K}\right]}^{-1}. \end{array}$$

One-step prediction error variance matrix

(6) $$\begin{array}{c} P_{k,k-1}=\phi_{k,k-1}P_{k-1}{\phi_{k,k-1}}^{T}. \end{array}$$

Estimated error variance matrix

(7) $$\begin{array}{c} P_{k}=\left[I-K_{k}H_{k}\right]P_{k,k-1}{\left[I-K_{k}H_{k}\right]}^{T}. \end{array}$$

The system uses a fusion reset structure, so there are

(8) $$\begin{array}{c} \left\{\begin{array}{c} \beta_{1}=\beta_{2}=\beta_{3}=\beta_{4}=\frac{1}{4},\\ \beta_{m}=0. \end{array}\right. \end{array}$$

Reorganize the data of the entire system according to the formula

(9) $$\begin{array}{c} Q^{-1}=Q_{m}^{-1}+\overset{n}{\underset{i=1}{\sum }}Q_{i}=Q^{-1}\beta_{m}. \end{array}$$

In the above formula, *Q* represents the data collection of the entire system. The system data satisfies the information conservation criterion in the process of reorganization; that is, the amount of data information before and after the reorganization is equal. If there is no correlation between the output of the subfilter and the main filter, the fusion is carried out according to the following formula:

(10) $$\begin{array}{c} \left\{\begin{array}{c} Xg=Pg\left[P_{m}^{-1}Xm+\overset{n}{\underset{i=1}{\sum }}\right],\\ Pg=\left[P_{m}^{-1}+\overset{n}{\underset{i}{\sum }}P_{i}^{-1}\right]. \end{array}\right. \end{array}$$

In the above-mentioned joint filter, the main filter continuously feeds back information to the subfilters, to realize the real-time update of the fusion data and improve the real-time and accuracy of the system filtering process. Data fusion can be divided into nonfeedback fusion systems, as shown in Figure 2.

There are also feedback fusion systems, which are based on the distributed nonfeedback fusion system. The fusion center was added to each feedback channel, as shown in Figure 3.

### 2.3. Student Constitution

Constitution refers to the human body acquired on the basis of genetic diversity and relatively stable characteristics in morphology and function. Physical strength is closely related to genetics, environment, nutrition, and exercise. Heredity only provides the precondition of physical status and development, and the strength of physical strength depends on the acquired environment, nutrition, health, exercise, and other factors. Therefore, scientific exercise and reasonable diet and nutrition are the most effective means to improve physical strength [6].

The physical problems of young people are related to the future of the country. The healthy growth of young people has laid a solid foundation for the development of the country. As can be seen from the numerous research results in recent years, the physique of young people has always been concerned. Many research results have carried out detailed investigations on the obesity problem of young people in urban areas, but few studies have been conducted on the health status of young people in rural areas, which account for the majority of China's population.

### 2.4. Influence of Aerobics on Physical Fitness

Aerobic exercise has a great influence on the improvement of students' physical fitness. Aerobic exercise refers to the ability to fully absorb oxygen in the body at any time during exercise. There are various types of aerobic exercise, such as swimming, jogging, aerobics, dancing, and cycling. It can be seen from the relevant research that aerobic exercise has physiological aspects. Body mass index, muscle strength, muscle endurance, increased muscle weight, cardiopulmonary endurance, and waist-to-hip ratio were improved. In addition, it can adjust your physical ability, help digestion, improve sleep quality, and strengthen physical function, mental function, and sports learning [7, 8].

Aerobics helps to consume energy, enhance physical strength, and improve health. The advantages of blood biochemical value have also been improved. The reduction of cholesterol, triglycerides, and low-density lipoprotein; the improvement of physiological metabolism; and the beautification of muscles can strengthen the antioxidant defense ability and other effects. For people with joint injuries or problems, aerobics training can enhance the angle of bones, muscles, and joints. Therefore, people who have problems with bones and joints can start with aerobic exercise that does not affect them. Life is a safety risk. Aerobics can be used to reduce the risk of exercise; aerobics will affect health. At the physiological level, aerobics training can improve physical strength and physiological and metabolic functions, strengthen antioxidant defense capacity, beautify muscle lines, and promote the strength of bone and muscles [9].

### 2.5. Relationship between Sports, Nutrition, and Physical Fitness

#### 2.5.1. Sports and Physique

Immunity is an important part of human body function to maintain health. We must fully understand the internal relationship between exercise and physique and analyze the physical ability to adapt to the external environment, so that people can use reasonable exercise or nutrition intake to adjust the immune state and maintain a healthy physique. Sports may change the immune function of the human body. The change of antibody ability produced by the human body after exercise will kill the bad cells, change the cell structure of the body, and affect the change of overall physical strength. However, we need to pay attention to the intensity management of physical exercise. Moderate exercise may improve people's immunity, but high-intensity physical exercise may have adverse effects, only to achieve the purpose of sports, to form a healthy function [10]. The purpose of exercise is not to harm oneself. Only by grasping the regular exercise method and performing sports appropriately can the purpose of exercise be achieved or a healthier body.

#### 2.5.2. Nutrition, Collocation, and Physique

Nutrition is the human body's need to maintain life and health, ensuring the body's growth and development, physical activity, and learning thinking. It must continue to ingest the necessary nutrients from food. Only a reasonable combination and intake of these nutrients can maintain normal life activities and physical health. The human body contains nutrients such as protein and vitamins, which will affect the body's immune function, which will affect the normal activity and exercise ability of the body. Protein is one of the essential nutrients for the human body. If protein intake is insufficient, the number of human cells and food cells will be reduced, and the function and ability of site chain proteins will be decreased. The characteristic of hyposecretion of synthetic substances is related to human diseases. The increase of probability will affect the normal function and action of the human body [11].

### 2.6. Influence of Sports and Nutrition on Students' Physique

#### 2.6.1. Regulate Body Function and Immunity

Physical strength of the human body is closely related to function and movement. The relationship between exercise and immunity is valuable. Therefore, to improve body function, students must pay attention to the important value of body movement. Using proper intensity exercise can not only improve the body's build and function but also make the shape of the body more standard. It can also strengthen the adjustment and improvement of the body organ system, which is beneficial to the improvement of students' body immune function. An important role is that the frequency and intensity of sports activities will affect the immune status of students. Because in sports, too high a rating will lead to a rapid decline in physical strength, thereby reducing immunity; and too high intensity may damage the body and cause harm to the body. In addition to reasonable intensity exercise, scientific intake of nutrition may also affect immune function. Medical research shows that intake of sugar, vitamins, and proteins can regulate immunity through the endocrine pathways, reduce the impact of students' exercise, and strengthen immunity. Stress is more convenient than nutrition. Nutrition can improve their own function and ensure the healthy development of immune function and physical ability [12, 13].

#### 2.6.2. Enhance the Students' Body Movement Ability and Defense Ability

The imbalance of students' diet structure and nutrient intake is a way for students to improve their body function through nutrition matching. Therefore, students must pay attention to the effect of exercise on physical strength. Proper intensity of exercise can adjust the body function. The most direct benefits of physical exercise are improved function of the heart and lungs. Through exercise, we can adjust the capacity and vital capacity of the respirator system, improve the respiratory function and heart function of the lung, and improve the innate organ function through acquired efforts. Moreover, it has a cumulative effect on the students in the growth and development stage. When the human body exercises, the human body is in a negative oxygen state, metabolizes body energy in a short time, and produces different metabolic intensities under the influence of different amounts of exercise. Therefore, to protect the body, it is necessary to adjust the intensity and cycle of physical exercise, reasonably; metabolize in the normal range; and ensure the effect of exercise [14].

#### 2.6.3. Reduce the Incidence Rate of Disease Infection

Students' healthy life can be improved by some methods to ensure the adjustment of body function and the enhancement of immunity. First of all, students must complete the nutrition intake of three meals a day on time, eat more fruits and vegetables, eat less snacks and junk food, and exercise for two hours to ensure the effectiveness of body function. Second, we must ensure the time and quality of sleep, develop good sleep habits, and maintain a standard of 7-8 hours of sleep a day. In addition, it is necessary to reduce smoking and drinking habits and develop healthy living habits. Finally, to reduce the incidence of other diseases caused by hypertension, fatty liver, hyperlipidemia, diabetes, and obesity, it is necessary to control the body weight reasonably and reduce the intake of fat and other food causing obesity. Live a good life in the habit of that period; also, there is a need to pay attention to the intake of nutrients. For example, to supplement vitamins, take more fruits and vegetables, and eat fish to supplement protein, so that the body's nutrients are more balanced, strengthen the body's immune function, and resist the impact of infection [15].

## 3. Aerobics Training and Nutrition Matching Experiment

### 3.1. Subjects

In this experiment, a total of 80 students from grade one of the key middle schools in our city were selected. The guidance of aerobics is the same. Each class teaches aerobics twice a week, and the guidance time of each aerobics is 45 minutes, a total of two and a half months, and 10 weeks of experimental time.

### 3.2. Experimental Test

The test time is divided into two stages: before and after the experiment, to ensure the accuracy of the test, the interval between the test before the test and the test after the test should not exceed 2 hours, so that the test should be performed immediately before the test and immediately after the test. To avoid the interference between the test items, the test time will be divided according to the exercise intensity of the test items. The examination time is arranged in the afternoon between the big class and the freshman. Pupils have a rest every weekend, and the exam time is from Monday to Friday.

### 3.3. Test Method

#### 3.3.1. Physical Fitness Test

In the physical test, choose to sit forward and do long jump, 50 m race, and 800 m run. This can reflect the physical level of students, such as flexibility, strength, agility, coordination, speed, and endurance. All students taking the exam must be in a state of health and free from hereditary diseases. During the test, sports shoes and sportswear must be worn. Do not wear nail shoes during the test. In the outdoor test project, the wind must be blown in case of adverse wind. Sit forward: held in the physical test room of Suqian Middle School. The students sit in the designated position with their heels closed and press the bending baffle at the front. When the students are ready, put their hands together and push the cursor forward to the farthest position. During the test, the knees of both feet must be kept straight. In a state of integrity, there are two opportunities for students to take the exam. The staff kept 1 place below the decimal point as 25.6 cm and recorded the farthest result.

1. One minute sit-up: students sit on their backs in the test room with their feet slightly away and knees bent about 90 degrees. Cross the back of the head with two fingers, and press the ankle with the other finger to fix the lower limb. Candidates need to sit with their elbows touching their knees and the shoulder blades lying on their back. After the pen sends out “start,” the instrument starts to record and stops after a minute, and the staff starts to count
2. Standing long jump: students participating in the test must wear sports shoes and sportswear. After the take-off point, the students will open 2 feet in parallel, preswing their arms properly, jump forward and up, and bend their knees to relax the cushion after landing. Once stabilized, move forward from the test area. Three times each test, select the best performance record, and keep 1 digit below the decimal point
3. 50 m: the students in the exam make two pairs and start standing at the starting point of 50 m. After listening to the starter's “preparation” instruction, the students' front and back feet open and become forward leaning. The starter swings down and sends out a “run” command. Mark, the students of the examination will go forward immediately after hearing the “execute” command. The timekeeper started the time when he saw the start of the flag. When the student's body passes the drop surface of the 50 m finish line, the clock will stop and record the student's 50 m run. A fraction of 50 meters is recorded to one place below the decimal point. The second place is to record the score according to the principle of “0” and not entering 1
4. 800 m: 16 student groups took the test, and each student had a digital shirt lined up at least 30 cm from the starting line of 800 m. All students in the examination begin with standing. After listening to the “carry out” instruction, the students ran along their trucks. You can split a track into a single track with a straight track. If you feel uncomfortable, you can abort the test for the next supplementary test. After the students finish 800 meters, students should not stop or sit but walk slowly along the inertia. When the flag was waving, the clock started, and the clock stopped when the student's body passed the vertical of the 800-meter finish line. The 800-meter fraction is recorded with one digit below the decimal point, and the two digits below the decimal point are recorded according to the principle of entering 1 other than “0” (3 minutes 55 seconds is changed to 235.2 seconds by computer input)
5. Height: the staff adjusted the height and weight in advance. The students were standing on the floor of the height and weight scale with their socks on their backs and their heels sticking together and leaving their feet at an angle of about 60 degrees. I kept my feet in the exam, straight arms close to pants, head and torso straight, looking forward, eye sockets, and upper ears at the same height. Staff confirmed that the student's scapula, fairy bone, and heel were close. When the line-up and test students meet the above requirements, the staff activates the start button, the horizontal pressure plate automatically drops to the head of the test students, the height of the students is automatically displayed, and the staff makes records
6. Weight: staff adjusted the height and weight of the testing machine in advance. Students are requested to wear uniforms, not decorations. Let the body stand upright as the student behavior of the examination. After maintaining a stable state, the staff presses the start button, and the examinee can exit after hearing the voice of “end of the examination.” The weight will be displayed automatically, and the staff will record it
7. Sebum thickness: the staff (female) adjusted the sebum examination apparatus in advance and selected three parts of the student's thigh, abdomen, and arm. The error is within 5% or 2 mm. The results are valid. In addition, the test is repeated. Abdomen: select the 2 cm right part of the student's navel button. The measurement method is the same as that of thigh examination. Arm: to naturally test the student's arm sag, select the midpoint connection between the acromion of the triceps of the upper arm and the elbow of the student's arm

#### 3.3.2. Physical Function Test

1. Vital capacity: the staff adjusted the vital capacity measuring machine in advance and trained the students in the method of vital capacity measurement and test. During the test, students must keep a relaxed and natural standing state. To exhale slowly, aim at the mouth until the breath cannot continue. The data will be displayed automatically. Two measurements will be made in total to get the best results. The interval between the two tests is within 15 seconds
2. Step test: the staff adjusted the height of the step to 35 cm and carried out the step experiment training for the students. Students move the steps up and down according to the rhythm of the metronome (120 beats/min) to make sure that the steps are consistent with the rhythm of the metronome. Students' left and right feet are tested alternately. Do not bend your upper body and knees when stepping on your feet. Keep a straight posture. After the test, the test students sit in the designated area, and the staff will measure the pulse of the test students in 1 minute~1:30 seconds, 2 minutes~2:30 seconds, 3 minutes~3:30 seconds. Evaluation index of step test = duration of step climbing (s) × 100/(2 × sum of 3 pulses during recovery)

### 3.4. Training Process

In the experimental 10-week aerobic exercise education, female students of grade one study and train physical exercise twice a week. In addition to the twice weekly aerobic exercise education, we only used the individual interview after the experiment, which had no impact on the study and life of 80 female students, to understand the activities outside the experimental time and judge the impact on the experiment. After 18 weeks of aerobics research, the height, weight, vitality, sebum, flexion, abdominal muscles for 1 minute, vertical jump, 50 m, 800 m, etc. of the first grade girls were tested to collect the choice of aerobics.

### 3.5. Data Collection

Due to the large amount of data, the experimental data obtained in this article are analyzed by statistical software and will not be repeated here. This article uses SPSS17.0 to collect statistics on students' body side performance and then uses data fusion technology to process and analyze the statistical data information through computer-assisted methods, optimize and integrate, complete decision-making and estimation tasks, and provide students' body side achievements to provide accurate information support.

## 4. Influence of Aerobics and Nutrition on Students' Physique

### 4.1. Influence of Aerobics Training Course on Students' Body Shape Indexes

Table 1 shows the comparative analysis of body shape indexes of students before and after aerobics training (*n* = 80).

It can be seen from Table 1 that height is mainly affected by the factors that are born. Among the main reasons for obtaining height, living environment, nutrition, diet, and exercise also have a certain influence on height. According to the comparative analysis of the body shape index of the first grade girls before and after the aerobics course selection in Table 1, after 10 weeks of aerobics training, the average height of the first grade girls increased by 1.19 cm. Aerobics is helpful to the growth of height. Proper exercise can promote the growth hormone secretion of female high school students. Growth hormone promotes the formation of cartilage at the end of bone and promotes the growth of bone end and cartilage, thus increasing the body. The height of the first grade girls without aerobics in Suqian Middle School is slightly lower than the national average height of the first grade girls, and the average height after aerobics is higher than the national average height of the first grade girls. It was shown that aerobics are beneficial to the increase of height of first grade girls, but the increase is not significant.  Figure 4 shows the BMI index evaluation table of female students in the senior one before and after aerobics training.

It can be seen from Figure 3 that the basis for measuring body weight and health is body mass index (BMI) = body weight (kg) × height^2^ (m). Before the experiment, the BMI of normal girls was 46.1%, that of lean type was 24.1%, that of obesity was 12.4%, that of obesity was 10.7%, and that of extreme obesity was 6.7%. After 10 weeks of aerobics training in Suqian Middle School, the normal BMI of female students in grade one was 55.1%, 22.1% thinner, 9.4% overweight, 7.7% obesity, and 5.7% obesity. The average BMI of the first grade girls in China was 47.1%, 23.8% thin, 12.2% fat, 10.4% obese, and 6.5% extremely thick.

The weight of female students who chose aerobics in grade 1 changed after training. The average weight decreased by 1.17 kg, and the relative weight changed. 45 minutes by calculating the exercise time of aerobics class students in Suqian Middle School, female high school students practice aerobic exercise for more than 30 minutes, and the rest time becomes shorter. Aerobics is an aerobic exercise. The main method of metabolism is the supply of aerobic energy. Girls in grade one take more than 30 minutes of aerobics. The body mainly consumes the energy supplied by fat to reduce body fat. Before the aerobics survey, the weight of the first grade girls was slightly heavier than the average weight of the domestic first grade girls, but after four and a half months and 18 weeks of aerobics, the weight of the first grade girls decreased to different degrees. Long-term high-intensity aerobics can effectively inhibit students' weight gain and can reduce a little.

### 4.2. Analysis of the Influence of Aerobics Training on Students' Physical Fitness Index

Physical strength can reflect the basic sports ability of girls. In the national physical fitness test, the girls were selected for bending position, one minute clamp, 50 m, and 800 m. Through these five tests, we can roughly reflect the flexibility, strength, speed, agility, endurance, and other qualifications of female high school students. For example, Table 2 is the comparative analysis table of female students' physical fitness indexes before and after aerobics training (*n* = 80).

According to the comparison and analysis of aerobics before and after (Table 2), the average level before the experiment increased from 13.78 cm to 17.24 cm, and the flexion index increased after 10 weeks of aerobics. In the training of aerobics, flexibility is needed for kicking, swinging, jumping, and horizontal collisions. When aerobics teachers teach aerobics to improve girls' softness and agility, they use soft training. Long-time aerobics can coordinate muscles and improve the flexibility of joints and ligaments. The flexibility, agility, and coordination of female senior high school students have been improved, which has a very obvious impact on the performance improvement of girls in sitting posture.  Figure 5 shows the indexes of students' physical fitness before and after aerobics training.

It can be seen from Figure 4 that after 10 weeks of aerobics exercise, one-minute abdominal muscle exercise increased from 23.9 before the experiment to 31.2. This is a big improvement. That is because after the training of aerobics, the waist and abdomen muscle strength and body coordination in girls has been an effective exercise, so there has been an effective development in the waist and abdomen muscle and coordination. The average standing long jump increased from 164.4 cm to 174.6 cm, and the standing long jump performance of girls was greatly improved. Standing long jump may reflect the strength of students' lower limbs and the coordination ability of the upper limbs and lower limbs. Aerobics includes walking, running, jumping, and other activities. After the fitness exercise, it can greatly improve the leg muscle strength.

Before the experiment, the results of 50-meter women were the same as the national average level of 50-meter women in grade 1. After 10 weeks of aerobics, the 50-meter running performance changed from 9.7 seconds to 9.5 seconds. The 50-meter run was 0.2 seconds faster. A 50-meter run can reflect a girl's speed, explosiveness, agility, reaction, and other qualities. This shows that bodybuilding helps to improve girls' speed ability. Aerobic exercise, including walking, running, jumping, and other activities; after aerobics, the muscles of the upper limbs and lower limbs can greatly improve the muscle strength of the waist and abdomen. It is beneficial to maintain the balance ability of the body when driving at high speed. The forward tilt angle of the body is effectively changed, and the final step length is increased. Strengthening the upper and lower limbs is helpful to improve the running ability of 50 m. After the step length and moving ability of kicking and swinging are effectively improved, the driving performance of 50 m is improved.

Before the experiment, women's 800 m performance was slightly lower than the national average level of female students in grade 1 in 800 m running. After 10 weeks of aerobics, the average performance of 800 meters changed from 253.2 seconds to 249.3 seconds, and the performance of 800 meters became 2.9 seconds faster. The 800-meter race reflects the function of the cardiovascular system, respiratory system, and muscle endurance of students. It is easy to have dyspnea in the 800-meter running test. Most of the girls who cannot bear the pressure of the chest are not very athletic. Their lower limbs are very heavy, and their movements are slow and nauseous. For students, it will stimulate the body, and it is easy to have muscle pain the next day. The 800-meter race is a national fitness test that girls have most. After 10 weeks of bodybuilding, the girl's cardiopulmonary function was improved. Over 800 meters, it can recover faster than before. The girl's performance and fear of the 800 m have been effectively improved.

### 4.3. Analysis of Students' Diet and Nutritional Status

Figure 6 shows the statistical chart of students' snack intake.

According to the statistics shown in Figures 6, 70.4% of freshmen's favorite snacks are desserts, fried foods, and seafood, which are 70.4%, 51.9%, and 52.6%, respectively. In addition to vinegar pickled food, students' preference for other snacks was more than 40%.

Among teenagers, the problem of snacks is widespread. It is well known that unscientific snack behavior hinders the growth and development of students. Malnutrition and other diseases can also pose health risks. In addition, most teenagers drink drinks such as water, and their daily intake of water is much less than the body needs, so it has a subtle impact on health for a long time. Therefore, it is essential to correct the unscientific diet life, establish the correct diet concept, and guide the students to improve their nutrition and health awareness.

### 4.4. Analysis on the Influence of Aerobics and Nutrition Balance on Students' Comprehensive Physical Quality

Figure 7 shows the influence of aerobics and balanced nutrition on comprehensive physical quality.

The data were analyzed and evaluated after fusion; it can be seen from Figure 6 that in the control group, without physical exercise and irregular diet, the comprehensive physical quality of the experimental subjects fluctuated on and off the standard line, and their physical condition was poor. After aerobics training, the physical fitness and other factors have been improved in the training process. In the experimental group with balanced diet and good nutrition, the physical quality is also relatively good. In the group with both aerobics training and nutrition balance, the overall physical quality changes significantly and the effect is better.

## 5. Conclusion

In this paper, the characteristics of aerobics, sports, and nutrition strategies are studied with the human body recognition technology of depth images. With a good nutrition strategy, the effects of aerobics exercise can be effectively improved. By analyzing the characteristics and movements of aerobics, using the standard template of aerobics exercise, in the daily exercise of aerobics, comparing the action with the template, you can better correct your own shortcomings and mistakes; combining the data in the analysis of the influence of aerobics training and nutrition on the physical indicators of the students, the analysis of the impact of the indicators of the physical fitness of the students, the analysis of the daily diet and nutritional status of the students, and the analysis of the impact of the comprehensive physical fitness of the students, a more accurate result can be obtained, for evaluation and analysis. The students are in the dual development stage of nutrition and intelligence. Ensuring the comprehensive nutrition of diet is the basis of all aspects of students' development. After investigating the nutrition and health status of all students in this school, it is found that there are some problems, such as physical discomfort, unreasonable diet, partial solar eclipse, unbalanced diet, and not paying attention to breakfast. Therefore, the government and schools should increase the interest of nutrition and health education for senior high school students and jointly deal with the nutrition and health problems of young people.

## Figures and Tables

**Figure 1:** Kalman filter (KF) algorithm.

**Figure 2:** Nonfeedback fusion system.

**Figure 3:** Fusion system feedback.

**Figure 4:** Body mass index evaluation table of female students in the senior one before and after aerobics training.

**Figure 5:** Physical fitness index of students before and after aerobics training.

**Figure 6:** Statistical chart of snack intake. Note: (a) Desserts (ice cream), (b) fried foods, (c) puffed foods, (d) instant noodles, (e) canned, (f) biscuits, (g) pickled foods (ham sausage), and (h) preserved fruits.

**Figure 7:** The influence of aerobics and nutrition balance on comprehensive physical quality.

**Table 1:** Comparative analysis of body shape indexes of students before and after aerobics training.

Test indicators	Before training	After training	Average value
Height (cm)	161.05 ± 12.45	162.36 ± 12.27	161.38 ± 11.24
Weight (kg)	55.53 ± 7.43	54.32 ± 6.17	55.14 ± 6.22
BMI index	21.4 ± 2.72	20.1 ± 3.03	21.2 ± 2.35

**Table 2:** Comparative analysis of female students' physical fitness indexes before and after aerobics training (*n* = 80).

Index	Before training	After training	Average value
Sitting forward flexion (cm)	13.78 ± 5.25	17.24 ± 4.28	13.54 ± 5.46
1 minute sit-ups	23.9 ± 5.2	31.2 ± 4.5	22.7 ± 5.4
Standing long jump (cm)	164.4 ± 12.5	174.6 ± 10.5	161.2 ± 12.8
50 m (s)	9.7 ± 1.5	9.5 ± 1.2	9.6 ± 1.4
800 m (s)	253.2 ± 41.2	249.3 ± 32.4	252.4 ± 40.2

## Data Availability

The data underlying the results presented in the study are available within the manuscript.

## References

[1] Hoelscher D. M., Moag-Stahlberg A., Ellis K., Vandewater E. A., Malkani R. (2016). Evaluation of a student participatory, low-intensity program to improve school wellness environment and students' eating and activity behaviors. *International Journal of Behavioral Nutrition and Physical Activity*.

[2] Basso-Vanelli R. P., Pires V. A., Lorenzo D., Labadessa I. G., Regueiro E. M. G., Costa D. (2016). Effects of inspiratory muscle training and calisthenics-and-breathing exercises in COPD with and without respiratory muscle weakness. *Respiratory Care*.

[3] Hu M., Zhong Y., Xie S., Lv H., Lv Z. (2021). Fuzzy system based medical image processing for brain disease prediction. *Frontiers in Neuroscience*.

[4] Ding S., Qu S., Xi Y., Wan S. (2020). Stimulus-driven and concept-driven analysis for image caption generation. *Neurocomputing*.

[5] Shan P. F. (2018). Image segmentation method based on K-mean algorithm. *EURASIP Journal on Image and Video Processing*.

[6] Abdulsalam N., Condrasky M., Bridges W., Havice P. (2017). The promise of andragogy and experimental learning to improve teaching of nutrition concepts to culinary arts students. *Journal of Food ence Education*.

[7] Gezer-Templeton P. G., Mayhew E. J., Korte D. S., Schmidt S. J. (2017). Use of exam wrappers to enhance students’ metacognitive skills in a large introductory food science and human nutrition course. *Journal of Food Science Education*.

[8] Tasker T. Q., Herrenkohl L. R. (2016). Using peer feedback to improve students' scientific inquiry. *Journal of ence Teacher Education*.

[9] Hamman S. T., Hopkinson K. M., Markham R. L., Chaplik A. M., Metzler G. E. (2017). Teaching game theory to improve adversarial thinking in cybersecurity students. *IEEE Transactions on Education*.

[10] Asada Y., Hughes A. G., Read M., Schwartz M. B., Chriqui J. F. (2017). High school students' recommendations to improve school food environments: insights from a critical stakeholder group. *Journal of School Health*.

[11] Lawson T. J., Blackhart G. C., Gialopsos B. M. (2016). Using the power balance wristband to improve students' research-design skills. *Teaching of Psychology*.

[12] Krustrup P., Dvorak J., Bangsbo J. (2016). Small-sided football in schools and leisure-time sport clubs improves physical fitness, health profile, well-being and learning in children. *British Journal of Sports Medicine*.

[13] Chang Y. C., Wang J. D., Chen H. C., Hu S. C. (2017). Aerobic-synergized exercises may improve fall-related physical fitness in older adults. *The Journal of Sports Medicine and Physical Fitness*.

[14] Meier N. F., Lee D. C., Sui X., Blair S. N. (2018). Physical activity, cardiorespiratory fitness, and incident glaucoma. *Medicine & Science in Sports & Exercise*.

[15] Kirkham A. A., Klika R. J., Ballard P. D. T., Downey M. P. (2016). Effective translation of research to practice: hospital-based rehabilitation program improves health-related physical fitness and quality of life of cancer survivors. *Journal of the National Comprehensive Cancer Network: JNCCN*.

